This article has been retracted.

# Targeted Nursing Combined with Endoscopic Submucosal Injection of Carbon Nanoparticles in the Treatment of Colorectal Cancer

**DOI:** 10.1155/2022/8663645

**Published:** 2022-05-31

**Authors:** Libo Yin

**Affiliations:** Department of Endoscopy, The First Affiliated Hospital of Shandong First Medical University, Jinan, Shandong, China

## Abstract

**Aim:**

To evaluate the effectiveness of targeted nursing in an endoscopic submucosal injection of carbon nanoparticles to locate colorectal cancer.

**Methods:**

From September 2017 to September 2019, 82 patients with colorectal cancer who underwent endoscopic submucosal injection of carbon nanoparticles for locating the tumor were recruited and assigned via the random number table method (1 : 1) to receive either conventional nursing (control group) or targeted nursing (observation group). Outcome measures included psychological status, compliance, nursing satisfaction, quality of life, and daily living ability.

**Results:**

After intervention, the self-rating anxiety scale (SAS) scores and self-rating depression scale (SDS) scores were decreased in both groups, with lower results in the observation group (*P* < 0.001). Patients given target nursing were associated with higher compliance and nursing satisfaction of patients versus conventional nursing (*P* < 0.05). Patients receiving targeted nursing had a better quality of life versus those receiving conventional nursing (*P* < 0.001). Targeted nursing resulted in a higher Barthel index (BI) in patients versus conventional nursing 1 d, 7 d, and 14 d after nursing (*P* < 0.05).

**Conclusion:**

Targeted nursing alleviates the negative emotions of patients with colorectal cancer and improves their compliance, nursing satisfaction, daily living ability, and quality of life.

## 1. Introduction

Colorectal cancer is a common malignancy with a high incidence [1]. Symptoms of colorectal cancer at the advanced stage include abdominal pain, constipation, and hematochezia, which severely compromise the quality of life of patients [2]. Laparoscopic surgery is widely used in the treatment of colorectal cancer. However, this surgery fails to accurately locate the lesion under the laparoscope. Tumors of small size can be accurately located under the laparoscope by injecting carbon nanoparticles nearby the lesion via endoscopy [3]. Patients with colorectal cancer may develop negative emotions, and conventional nursing is ineffective in ameliorating their psychological status, resulting in compromised treatment compliance and quality of life [4]. Targeted nursing can relieve patients' negative emotions such as anxiety and improve the quality of life and nursing satisfaction [5]. Studies have shown that traditional Chinese medicine (TCM) treatment of colorectal cancer has shown unique advantages in alleviating symptoms, increasing survival rate, improving quality of life, enhancing physical fitness, and reducing toxic side effects of radiotherapy [6, 7]. Clinically, surgery and chemotherapy are the mainstay of treatment to maximally eliminate tumor cells and reduce tumor recurrence and metastasis. Surgery, chemotherapy, and radiotherapy are the current standard modes of comprehensive treatment for colorectal cancer in Western medicine, which impair the immune function of patients to some extent and compromise their prognosis. The TCM treatment, Fuzheng Peiben decoction, can be used to strengthen the patient's immune status. In the present study, 82 patients with colorectal cancer who underwent endoscopic submucosal injection of carbon nanoparticles for locating the tumor were recruited to evaluate the effectiveness of targeted nursing in endoscopic submucosal injection of carbon nanoparticles to locate colorectal cancer.

## 2. Materials and Methods

### 2.1. General Materials

From September 2017 to September 2019, 82 patients with colorectal cancer who underwent endoscopic submucosal injection of carbon nanoparticles for locating the tumor were recruited and assigned via random number table method to receive either conventional nursing (control group, *n* = 41) or targeted nursing (observation group, *n* = 41). There was no statistical difference in patient characteristics between the two groups (*P* > 0.05) (Table 1). The research was approved by the Ethics Committee of the First Affiliated Hospital of Shandong First Medical University, no. SD97719.

### 2.2. Inclusion and Exclusion Criteria

Inclusion criteria were as follows: patients who met the diagnostic standard for colorectal cancer [6], who were diagnosed with colorectal cancer by CT or MRI, who were treated with the endoscopic submucosal injection of carbon nanoparticles localization, and who provided undersigned informed consent. Exclusion criteria were as follows: patients with other tumors, with infections, with heart, kidney, and liver dysfunctions, with a history of mental illness, and with low treatment cooperation.

### 2.3. Methods

#### 2.3.1. Control Group

The control group received conventional nursing, including health education, medication instruction, and routine cleaning.

#### 2.3.2. Observation Group

The observation group received targeted nursing. (1) Health education: patients were given relevant knowledge of colorectal cancer, such as its causes, clinical manifestations, treatment methods, and the purpose, procedures, significance, risks, and related precautions of surgical treatment to increase patients' awareness of the disease. (2) Psychological nursing: the nurses actively communicated with the patients to help them maintain a positive attitude and enhance patient self-confidence. (3) Physical nursing: the patients were instructed to perform muscle relaxation and breathing exercises. During training, the patients were instructed to perform abdominal breathing for 5–10 minutes, thrice daily. (4) Medication nursing: the medicines should be strictly checked to guarantee drug safety. The patients were supervised by the nurse during medication. (5) Diet nursing: the patients were instructed to follow a light and high-protein diet and were advised against spicy and irritating foods, which facilitated immunity restoration and robust postoperative recovery.

The patients also received Fuzheng Peiben decoction. The ingredients including 30 g of Astragali Radix, 6 g of Angelicae Sinensis Radix, 5 g of Panacis Quinquefolii Radix, 12 g of Atractylodis Macrocephalae Rhizoma, 30 g of Herba Patriniae, 30 g of Herba Hedyotidis, 30 g of Poria, 30 g of Chinese yam, 30 g of Semen Coix, 6 g of licorice root. 15 g of Bupleuri Radix, 10 g of Cyperi Rhizoma, and 10 g of tangerine peel were added for liver and spleen deficiency. 10 g of nutmeg and 10g of Evodiae Fructus were added for cold and dampness in the spleen and kidney. 20 g of Prunellae Spica and 30 g of Cremastrae Pseudobulbus; Pleiones Pseudobulbus were added for heat toxicity. 20 g of Asini Corii Colla was added for qi and blood deficiency. The above herbs were decocted with 500 ml of water in the automatic decoction machine, with the set at 120°C, decoction time of 1 h, and a pressure of 1.5–1.7 K. After decoction was completed, the liquid flowed to the automatic packing machine for vacuum packing, with 2 bags of 100 ml per dose.

### 2.4. Observation Indexes

1. Negative emotions: the self-rating anxiety scale (SAS) [7] was used for evaluation, in which severe anxiety was over 69 points, moderate anxiety was 60–69 points, mild anxiety was 50–59 points, and normal was less than 50 points. The self-rating depression scale (SDS) [8] was used for scoring, in which severe depression was over 72 points, moderate depression was 63–72 points, mild depression was 53–62 points, and normal was less than 53 points.
2. Compliance: it contained exercise compliance, medication compliance, and dietary compliance. Compliance rate = (complete compliance + partial compliance)/total numbers ×100%.
3. Nursing satisfaction: it was assessed according to the questionnaires designed by nurses with 8 items in total and five levels ranging from “highly satisfied” to “extremely dissatisfied.” Satisfaction rate = (highly satisfied + satisfied + average)/total numbers ×100%.
4. Quality of life: it was evaluated with the MOS 36-item short-form health survey (SF-36) scale [9], with a total score of 100 points. The score was proportional to the quality of life.
5. Daily living ability: the Barthel index (BI) [10] was used for the assessment of daily living ability 1 d before intervention, after intervention, 7 d after intervention, and 14 d after intervention, with a total score of 100 points. The higher the score, the better the ability.

### 2.5. Statistical Methods

This study used SPSS 23.0 for data analyses. The quantitative data are expressed as (‾*x* ± *s*) and analyzed using the *t*-test, with all the quantitative data conforming to normal distribution. The qualitative data are expressed as *n* (%) and analyzed using the chi-square test. The rank sum test was used to analyze the ranked data. Repeated measurement data were verified using analysis of variance (*P* < 0.05).

## 3. Result

### 3.1. Comparison of SAS Scores and SDS Scores

The SAS scores and SDS scores of the two groups before intervention were similar (*P* > 0.05). After intervention, the SAS scores and SDS scores were decreased in both groups, with lower results in the observation group (*P* < 0.001) (Table 2).

### 3.2. Comparison of Compliance

Targeted nursing was associated with higher treatment compliance (95.12%) of patients versus routine care (73.17%) (*Z* = 2.201, *P* = 0.028) (Table 3).

### 3.3. Comparison of Nursing Satisfaction

The observation group had a higher nursing satisfaction (97.56%) than the control group (80.49%) (*Z* = 2.262, *P* = 0.024) (Table 4).

### 3.4. Comparison of Quality of Life

Patients receiving targeted nursing had a better quality of life versus those receiving conventional nursing (*P* < 0.001) (Table 5).

### 3.5. Comparison of Daily Living Ability

Targeted nursing resulted in a higher Barthel index (BI) in patients versus conventional nursing 1 d, 7 d, and 14 d after nursing (*P* < 0.05) (Figure 1).

## 4. Discussion

The development of colorectal cancer is a multistep, multistage, and multigene process involving multiple genetic and environmental factors leading to colonic mucosal epithelial cell carcinogenesis, the mechanism of which involves uncontrolled cell proliferation and is related to the regulatory balance of apoptosis [10]. Recent research has shown that Fas/FasL may be involved in the immune escape mechanism in tumor development and in the countermeasure of tumor cells against killing by the body's immune cells [11]. The number of apoptotic cells decreases after colorectal epithelial cell carcinogenesis, and the disruption of apoptotic mechanisms is an important causative factor for cell carcinogenesis. The expression of Fas protein in hypofractionated colorectal cancer is lower than that in highly differentiated colorectal cancer, suggesting that the absence of Fas protein expression can reduce apoptosis and thus the imbalance between apoptosis and proliferation, resulting in accelerated cancer cell growth. FasL is commonly expressed in colorectal cancer with a higher frequency of expression than in initial nonmetastatic colorectal cancer, and the number of active T lymphocytes is greatly reduced.

About 60% of colorectal cancer locates at the junction of the rectum and the sigmoid colon and the rectum. It is a common gastrointestinal tumor and ranks the second among gastrointestinal tumors [11, 12]. Surgery is a common method of treatment for colorectal cancer. The efficacy of endoscopic minimally invasive treatment on colorectal cancer and its safety is promising [13, 14]. However, external factors and psychological factors may predispose patients to postoperative complications such as infections, which compromise the surgical results and aggravate their physical and mental pain [15]. With the development of modern medical technology, clinical treatment is no longer limited to improving the survival rate of patients but paying more attention to the quality of life [16].

Patients with colorectal cancer often experience negative emotions such as anxiety, fear, tension, and depression, resulting in poor sleep quality and treatment efficiency [17]. Specific psychological and emotional nursing contributes to relieving the negative emotions of patients, thereby improving their sleep quality and quality of life [18]. In the present study, the result showed that after intervention, the SAS scores and SDS scores were decreased in both groups, with lower results in the observation group, and patients receiving targeted nursing had a better quality of life versus those receiving conventional nursing. It is suggested that targeted nursing relieves patients' negative emotions and improves their quality of life. Targeted nursing is a new patient-centered nursing model, which provides patients with targeted nursing comprehensively throughout the entire process, especially in psychological and physiological aspects [19, 20].

The TCM decoction used in this study strengthens the spleen, benefits qi, and helps to restore the immune function of colorectal cancer patients. Astragali Radix enhances the phagocytic function of the reticuloendothelial system, significantly increases the number of blood leukocytes and polymorphonuclear leukocytes, elevates the phagocytic percentage and phagocytic index of macrophages, enhances the activity of natural killer cells (LAK) activated by lymphokine (interleukin-2), and promotes both humoral and cellular immunity. Its active ingredient F3 has been shown to have restorative effects on lymphocyte function in cancer patients in vitro and has been found to completely reverse the immunosuppression caused by cyclophosphamide in animal models in vivo, suggesting that the components of Astragali Radix may be a promising biological response modifier in immunotherapy. Ginseng has the effect of tonifying the middle and benefiting qi, generating fluid and harmonizing the stomach, and can significantly enhance the function of the reticuloendothelial system, which is even stronger when combined with Astragali Radix. This formula nourishes the middle Jiao, invigorates blood circulation, resolves blood stasis, eliminates symptoms and disperses nodules, and has a certain effect on malignant tumors in relieving cancer foci, which is related to the enhancement of immunity. It alleviates the damage of chemotherapy drugs on the liver, kidney, and nerves and has a significant effect on maintaining the function of the hematopoietic system.

## 5. Conclusion

In the present study, the result showed that targeted nursing resulted in a higher quality of life, BI, and treatment compliance versus routine care, indicating that targeted nursing improves patients' quality of life, daily living ability, compliance, and nursing satisfaction.

In conclusion, targeted nursing alleviates negative emotions of patients with colorectal cancer and improves their compliance, nursing satisfaction, daily living ability, and quality of life.

## Figures and Tables

**Figure 1:** Comparison of daily living abilities at different times. Compared with conventional nursing 1 d, 7 d, and 14 d after nursing,^*∗*^*P* < 0.05.

**Table 1:** Comparison of general materials.

Group	*n*	Gender		Average (years old)	Average course (years)
		Male	Female		
Observation group	41	22	19	58.14 ± 8.12	4.14 ± 1.24
Control group	41	23	18	59.34 ± 8.55	4.35 ± 1.11
*χ* ^2^/*t*		0.049		0.652	0.808
*P*		0.824		0.517	0.422

**Table 2:** Comparison of SAS scores and SDS scores (‾*x* ± *s*, score).

Group	*n*	SAS		SDS	
		Before intervention	After intervention	Before intervention	After intervention
Observation group	41	63.35 ± 5.14	43.58 ± 5.14^*∗*^	56.38 ± 5.41	44.39 ± 4.11^*∗*^
Control group	41	62.78 ± 5.46	54.29 ± 5.68^*∗*^	57.98 ± 5.63	53.87 ± 4.32^*∗*^
*t*		0.488	8.952	1.312	10.181
*P*		0.628	<0.001	0.193	<0.001

^*∗*^The comparison before intervention, *P* < 0.05.

**Table 3:** Comparison of compliance (*n*, %).

Group	*n*	Complete compliance	Partial compliance	Noncompliance
Observation group	41	23 (56.10)	16 (39.02)	2 (4.88)
Control group	41	16 (39.02)	14 (34.15)	11 (26.83)
*Z*			2.201	
*P*			0.028	

**Table 4:** Comparison of nursing satisfaction (*n*, %).

Group	*n*	Very satisfied	Satisfied	Normal	Dissatisfied	Extremely dissatisfied
Observation group	41	24 (58.54)	13 (31.71)	3 (7.32)	1 (2.44)	0 (0.00)
Control group	41	17 (41.46)	10 (24.39)	6 (14.63)	5 (12.20)	3 (7.32)
*Z*				2.262		
*P*				0.024		

**Table 5:** Comparison of quality of life (‾*x* ± *s*, score).

Group	*n*	Psychology	Emotion	Physical body	Society
Observation group	41	81.24 ± 7.35	86.57 ± 7.48	79.88 ± 7.44	82.45 ± 7.19
Control group	41	74.48 ± 6.95	76.98 ± 7.12	65.34 ± 6.15	70.51 ± 6.43
*t*		4.279	5.946	9.645	7.926
*P*		<0.001	<0.001	<0.001	<0.001

## Data Availability

The data generated or analyzed during this study are included within the article.
